This article has been retracted.

# Arthroscopic Anterior Cruciate Ligament Injury in Clinical Treatment of Joint Complications and CT Observation

**DOI:** 10.1155/2021/6667046

**Published:** 2021-02-22

**Authors:** Cheng Ji, Yuan Chen, Liulong Zhu, Jian Zhang

**Affiliations:** ^1^Affiliated Hangzhou First People's Hospital, Zhejiang University School of Medicine, Orthopedics Department, Hangzhou 310006, Zhejiang, China; ^2^Affiliated Hangzhou First People's Hospital, Zhejiang University School of Medicine, Anesthesiology Department, Hangzhou 310006, Zhejiang, China

## Abstract

Arthroscopy is the gold standard for diagnosing ACL injuries. It is a dual clinical technique for examination and treatment, which can effectively target the injury site for repair and treatment and can also accurately identify the lesion site and determine the degree of ligament injury through visual and three-dimensional observation of ligament injuries that are difficult to detect on imaging. However, this technique is invasive, so the clinic still needs to improve the related auxiliary imaging examination. In this paper, we performed MPR and VRT on patients with ACL injury and postprocessed the data. The diagnostic compliance rate of dual-source CT was 91.67% (33/36), the true positive rate was 93.33% (28/30), the missed rate was 6.67% (2/30), the true negative rate was 83.33% (5/6), and the misdiagnosis rate was 83.33% (5/6). The rate of true negative was 83.33% (5/6), and the rate of false diagnosis was 16.67% (1/6). Kappa analysis of the consistency between dual-source CT and arthroscopy showed a Kappa value of 0.719, indicating a high degree of consistency between the two examinations. In conclusion, MPR and VRT images are of clinical value for the diagnosis of ACL injury. In addition, dual-source CT can measure the CT value of the ACL and the thickness of each segment by MPR and VRT postprocessing techniques to diagnose the ligament injury in an objective, quantitative, and noninvasive way and can use dual-energy staining techniques to predict the ligament injury in a more intuitive way, which is not available in some arthroscopes.

## 1. Introduction

Knee injury is a common orthopedic disease, including meniscal injury, ligament injury, and other types, among which anterior cruciate ligament injury is more common. The anterior cruciate ligament of the knee is an important tissue to maintain the normal physiological activities of the knee joint, and once injury occurs, it can easily affect the stability of the knee joint structure, which can eventually lead to the limitation of the knee joint activities of patients. Patients with suspected ACL injuries need to be identified and diagnosed as early as possible, and treatment measures should be taken in a timely manner to reduce the degree of ACL injury and promote the recovery of the damaged ligament. Anterior cruciate ligament injury of the knee is a common and frequent disease in orthopedic surgery, and its injury mechanism is mostly due to excessive knee extension, knee flexion, external rotation, and internal rotation caused by external forces [1, 2]. Arthroscopy is the gold standard for the diagnosis of ACL injury [3], but because of its invasive operation, clinical diagnosis still needs to be made with the help of relevant imaging examinations. MRI is the preferred method of examination for ACL injury because of its clear display of ACL morphology and alignment [4], but it has the disadvantages of being time-consuming and contraindicated.

Dual-source CT [5–8] has a higher resolution of the ACL and more visualization of the ACL injury site and characteristics, and has the advantages of short time and few contraindications to examination [9]. Dual-source CT volumetric imaging can obtain MPR, VRT, and tendon staining of the ACL through postprocessing software, and the measured values can objectively reflect whether there is damage to the ligament, and it is an indispensable diagnostic method for the diagnosis of patients with combined fractures and other injuries. Compared with the invasive method of arthroscopy, the noninvasive imaging is more convenient and faster. In this paper, we investigate the value of dual-source CT imaging for the diagnosis of ACL injuries in the knee by combining anatomy with dual-source CT imaging and comparing arthroscopic findings. ACL reconstruction is one of the important methods to restore knee stability after ACL rupture [10, 11]. In the past decades, most patients with ACL rupture have undergone ACL reconstruction instead of conservative treatment [12]. However, because some studies in recent years have reported that ACL reconstruction is a risk factor for the development of knee osteoarthritis, which includes patellofemoral and tibial osteoarthritis, leading some patients to opt for conservative treatment [13, 14]. Essentially, the development of patellofemoral and tibial osteoarthritis after ACL rupture is caused by a combination of risk factors, such as altered knee biomechanics after reconstruction, knee cartilage damage, and meniscal damage [15]. As shown in Figure 1, there are various complications in surgery using joint reconstruction. Regardless of whether patients choose conservative or surgical treatment, approximately half of patients develop patellofemoral joint osteoarthritis on radiographic images 10–20 years after ACL rupture [16]. Moreover, patellofemoral osteoarthritis is often the most common and earliest manifestation of knee osteoarthritis after ACL surgery [17]. The development of knee osteoarthritis after ACL injury will seriously affect the quality of life of patients [18–20]. Although the exact mechanism by which patellofemoral osteoarthritis occurs after ACL injury is unknown, patellofemoral arthropathy is seen on MRI in approximately half of young adults in the first year after ACL reconstruction [21].

Of all knees with normal cartilage during ACL reconstruction, approximately half showed cartilage degeneration at the second arthroscopic examination 18 months after the reconstruction, and most occurred in the patellofemoral joint [22]. Because of the limited ability of articular cartilage to repair itself, it is often difficult to heal through self-repair after cartilage injury occurs. In recent years, with the continuous exploration and breakthroughs in cartilage repair by molecular materials, cell biology, and other disciplines, early intervention treatment of cartilage injury has gradually become possible. Moreover, patients undergoing ACL reconstruction are generally young and have high functional requirements for the knee joint, and the occurrence of patellofemoral joint osteoarthritis after ACL reconstruction will seriously affect the quality of life of patients [23]. Therefore, early diagnosis and intervention of patellofemoral joint cartilage injury are of great importance to prevent the occurrence and development of patellofemoral joint osteoarthritis in these patients [24].

Altered patellofemoral joint biomechanics may be a cause of patellofemoral joint osteoarthritis after ACL reconstruction. Although the biomechanics of the normal patellofemoral joint has been well studied, studies on the changes in cartilage loading of the patellofemoral joint in humans after ACL reconstruction have been rarely reported [25]. It was found that the patellar motion trajectory was not fully restored after single-bundle ACL reconstruction and remained significantly different compared to the healthy knee. These altered patellar motion trajectories may lead to altered patellofemoral joint contact biomechanics. Since normal cartilage mechanical loading is essential for cartilage development and maintenance, abnormal patellofemoral joint biomechanics may lead to patellofemoral joint cartilage degeneration, which may further lead to patellofemoral joint osteoarthritis. In some patients, local bleeding occurs after anterior cruciate ligament injury of the knee, resulting in a lack of contrast between the ligament and surrounding tissues, and the relatively low resolution of soft tissues on CT examination may lead to a missed diagnosis. Magnetic resonance examination has a higher soft tissue resolution compared with CT examination, and it can scan the patient's damaged area from multiple angles. The difference between magnetic resonance imaging of partial and that of complete tears of the anterior cruciate ligament of the knee is significant, so it has a clear advantage to identify whether the anterior cruciate ligament fibrin is intact more accurately.

## 2. Data and Methods

### 2.1. Research Subjects

Seventy-two patients who visited our orthopedic surgery department from January 2017 to September 2018 were included, including the experimental group, 21 males and 15 females, aged 20 to 51 years, with a mean age of (33.5 ± 10.8) years. In the comparison group, there were 21 males and 15 females, aged 22 to 55 years, with a mean age of (35.2 ± 12.5) years. All of them presented with unilateral knee discomfort and several symptoms (knee swelling, pain, unstable walking, limited flexion and extension activities, etc.) and positive signs such as anterior drawer test, Lachman test, and axial shift test. The initial diagnosis was unilateral anterior cruciate ligament injury. All patients who participated in this study had a full understanding of the purpose and procedure of the study before the experiment, and the patients agreed to perform dual-source CT and signed an informed consent form, which met the requirements of medical ethics and was approved by the ethics committee of our hospital. The patient was scanned with a dual-source Siemens 64-row CT machine in dual energy mode; the patient was placed in a supine position with both knees naturally extended and together; the scanning range was from the level of the superior border of the femoral condyle up to the level of the inferior border of the fibular head. The CTDICOM images of both knees were acquired, and the data were processed by postprocessing software for multiplanar reconstruction and dual-energy mode image processing to obtain MPR and VRT images. The general information of selected patients is as shown in Table 1.

### 2.2. Research Methods

A detailed preoperative history was taken and a physical examination was performed. After successful epidural anesthesia, a conventional arthroscopic surgical approach was performed. During the operation, the anterior cruciate ligament injury was carefully examined, the suspected injury site was explored, and we explored whether there were combined injuries in other areas, and the operation was recorded in detail.

MPR and VRT images: the high-voltage sequence in dual-energy mode was selected, and the multiplanar reconstruction module was chosen to reconstruct the bilateral ACL in coronal and sagittal positions (30 layers, 1 mm layer thickness, 0.5 mm layer spacing). The center of the ligament was the center point of the reconstructed localization image. Determination of the central level: the largest cross-section of the ACL was selected as the central level, and the region of interest (ROI) was drawn at the central level by an associate chief physician and measured numerically. Length measurement: the ACL was curved, so the curve measurement button was selected, and the value obtained was the full length of the ligament in millimeters (mm) along the midline of the ACL. Thickness measurement: the anterior-posterior distance of the ACL is measured in segments, divided into the beginning, middle, and end segments (parallel to the ACL), and the thickness of each segment is measured at the thickest point, which is the thickness value of the segment in millimeters (mm). Dual-energy staining mode: two sequences (high-voltage and low-voltage scanning sequences) in the dual-energy mode were selected and entered into the tendon module for multiplanar reconstruction (50 layers, 1.1 mm layer thickness, 0.5 mm layer spacing), with the center of the reconstructed image positioned at the center of the ligament.

### 2.3. Statistical Analysis and Results

The data were statistically analyzed using SPSS 22.0 statistical software. The diagnostic comparison between dual-source CT and arthroscopy for ACL injury was analyzed by the consistency test (Kappa). The values of MPR and VRT images of bilateral ACL were expressed as (*x* ± *s*) and analyzed by *t*-test, and *P* < 0.05 was considered statistically significant.

Of the 36 patients initially diagnosed with unilateral anterior cruciate ligament injury of the knee, 30 (18 men and 12 women) were diagnosed by arthroscopy. Eight patients had an injury at the beginning of the ACL, 13 patients had an injury at the middle segment, and 9 patients had an injury at the end segment. Using arthroscopy as the gold standard for diagnosis, Kappa analysis was performed between dual-source CT and arthroscopy, and the results showed that the Kappa value was 0.719, indicating a high degree of agreement between the two. The diagnostic compliance rate of dual-source CT was 91.67% (33/36), the true-positive rate was 93.33% (28/30), the missed rate was 6.67% (2/30), the true-negative rate was 83.33% (5/6), and the misdiagnosis rate was 16.67% (1/6). The CT values, lengths, and thicknesses of the ACL at the beginning, middle, and end points were statistically different between the healthy and the affected side of patients diagnosed with ACL injury by arthroscopy. The VRT and MPR images showed a hypodense area at the beginning of the ACL with blurred edges and no change in density at the middle segment; the thicknesses of the ligaments at the beginning and middle segments increased, but no significant change in ligament density was observed. There were no signs of fracture in the femur and tibia. The above suggests an injury to the anterior cruciate ligament initiation segment.

## 3. CT Observation of Complications of the Joint in Single Bundle Reconstruction of the Anterior Cruciate Ligament

### 3.1. Changes in Patellar Cartilage Thickness

With the results of this experiment, we found that the thickness of patellar cartilage after anterior fork ligament reconstruction was reduced compared to that before reconstruction, and the difference was statistically significant. This result is consistent with the results of previous studies. The use of MRI to measure cartilage thickness has been widely used in studies of knee osteoarthritis in the past. At 4-year follow-up of patients with knee osteoarthritis, thinning of tibial articular cartilage thickness correlated with the severity of knee osteoarthritis, and the development of knee osteoarthritis on radiographic images correlated with a decrease in cartilage thickness between the first 2 years and the second 2 years (OR = 1.3; OR = 3.4), while a decrease in cartilage thickness between the second 2 years correlated with an increase in clinical symptoms (OR = 1.5). A 1 mm reduction in articular cartilage thickness over 2 years is an important independent predictor of articular cartilage damage. Previous studies have found a high incidence of degenerative changes in the knee after ACL reconstruction, especially the development and progression of patellofemoral articular cartilage injury. In this experiment, we found that the average reduction in patellar cartilage thickness of 0.33 mm at 6 months after ACL reconstruction may be associated with the development and progression of patellofemoral cartilage injury and patellofemoral joint osteoarthritis after ACL reconstruction, as shown in Figure 2. Due to the complex structural and biomechanical characteristics of the knee joint, ACL injury will result in altered mechanical loading of the patellofemoral joint. Previous studies have demonstrated that the kinematic changes in the tibiofemoral joint associated with ACL injury result in a change in the relative elongation and orientation of the patellar tendon, and this biomechanical abnormality of the patellar tendon will result in altered patellofemoral cartilage contact and patellar motion trajectory, disrupting the normal mechanical loading of the patellofemoral joint. However, normal articular cartilage mechanical loading is critical for the development and maintenance of articular cartilage. It was found that patients with anterior fork ligament rupture had a mean reduction in femoral talocrural cartilage thickness of 0.88 mm 2 years after injury.

Stress deformation of patellofemoral cartilage in conservatively treated knees after ACL injury was greater than in the contralateral healthy knee, and patellofemoral joint thickness was thinner than in the contralateral healthy knee. Furthermore, the risk of patellofemoral cartilage injury increased 3-fold in the first year after ACL injury and 30-fold between 7 and 11 years after ACL injury. The above evidence suggests that ACL injury is often accompanied by a reduction in patellofemoral cartilage thickness and an increased risk of patellofemoral cartilage injury due to changes in patellofemoral joint biomechanics. BO, which assesses the lateral displacement of the patella, and PTA, which assesses the tilt angle of the patella, were reduced after ACL reconstruction compared with the prereconstruction period, but the differences were not statistically significant. This suggests that ACL reconstruction may have little effect on lateral patellar displacement and patellar tilt angle, and that biomechanical abnormalities of the patellofemoral joint may persist after ACL reconstruction. According to several previous studies, greater tibial external rotation excursion and cross-sectional rotational range of motion still exist in the knee after ACL reconstruction compared with the healthy knee.

These changes will affect the biomechanics of the patellar tendon, which will lead to changes in the biomechanics of the patellofemoral joint. Further studies have confirmed that the kinematic abnormalities of the patellofemoral joint due to ACL injury cannot be completely corrected after ACL reconstruction, mainly in the form of increased patellar external rotation, lateral tilt, and lateral displacement that remain after ACL reconstruction. Similarly, these abnormal patellofemoral joint biomechanics that cannot be fully corrected by ACL reconstruction may lead to patellofemoral cartilage degeneration. In some sports practitioners who underwent ACL reconstruction, it was found that the patellofemoral joint on the surgical side of these patients had greater pressure and compression than within the contralateral normal knee joint. Several previous publications have reported a reduction in patellofemoral cartilage thickness within the knee joint of the patient's surgical side after ACL reconstruction.

The results of this study are similar to our experimental results, which found that patellofemoral cartilage thickness was reduced after ACL reconstruction compared with that before reconstruction. Knee arthroscopy at year 1 after ACL reconstruction revealed significant deterioration of patellofemoral cartilage degeneration. The presence of patellofemoral cartilage damage at year 1 after ACL reconstruction predicted poor clinical function at year 3 after reconstruction. There is a high incidence of degenerative changes in the knee, particularly the development and progression of patellofemoral cartilage injury, within 5 years of ACL reconstruction. The above studies suggest that patients after ACL reconstruction continue to have patellofemoral joint biomechanical abnormalities that may be associated with patellofemoral joint cartilage degeneration and reduced cartilage thickness after ACL reconstruction.

### 3.2. Anterior Displacement of the Tibia Relative to the Femur

The increase in ISR to assess patellar height after ACL reconstruction may be due to a decrease in patellar tendon tension due to the anterior displacement of the tibia relative to the femur after an ACL tear, which can be observed on MRI of ACL injuries as the patellar tendon wave sign, which would result in a relative shortening of the measured patellar tendon length. After ACL reconstruction, the patellar tendon is no longer tortuous and shortened as the tibia is no longer anteriorly displaced, and the ISR increases after reconstruction as shown in Figure 3. Although patients with ACL injuries, whether treated conservatively or operated on as early as possible (within 2 months), have been found to have thinned femoral talocrural cartilage at 1-2 years' postreconstruction follow-up, newer studies have noted that patients who opted for surgical treatment after ACL injury had less reduction in patellofemoral cartilage thickness than those who opted for conservative treatment.

This may be because ACL reconstruction can partially restore the abnormal biomechanics of the patellofemoral joint. The anterior-posterior stability of the tibiofemoral joint improves after ACL reconstruction, and the tibial tuberosity moves posteriorly relative to the patellar tip, restoring the sagittal plane angle of the patellar tendon to a level similar to that of a healthy knee. Restoration of the sagittal plane angle of the patellar tendon reduces abnormal patellar flexion and restores normal proximal and distal cartilage contact of the patellofemoral joint cartilage because the inferior pole of the patella is no longer pulled forward relative to the femur. This demonstrates that ACL reconstruction has a protective effect on the patient's patellofemoral cartilage. Evidence from the above studies suggests that ACL injury will result in changes in patellofemoral joint biomechanics and that patellofemoral cartilage thickness decreases after ACL injury. Some of the patellofemoral joint biomechanical abnormalities may persist after ACL reconstruction. Although the reduction in patellofemoral cartilage thickness was delayed after ACL reconstruction, the reduction in patellofemoral cartilage thickness persisted after reconstruction. This is consistent with the experimental findings we observed. However, conservative treatment with delayed elective ACL reconstruction (within 2-3 years) after ACL injury was found to be better at reducing the reduction in patellofemoral cartilage thickness in patients with ACL rupture than early reconstruction (within 10 weeks). The mechanisms underlying the different cartilage damage under different treatment strategies are not known. It is possible that the prolonged duration of the intra-articular cellular inflammatory response in the knee caused by acute ACL injury or further activation of a new inflammatory response in response to surgical stimulation of ACL reconstruction may lead to cartilage degeneration and reduction of cartilage thickness in the patellofemoral joint. On the other hand, patellofemoral cartilage is the only cartilage that exhibits significant deformation during increased mechanical loading of the knee joint.

Therefore, during the rehabilitation exercise after ACL reconstruction, long-term inflammation under increasing mechanical load on the knee joint during the early recovery exercise phase may be closely related to the reduction of patellar cartilage thickness. According to previous studies, the thickness of knee cartilage is also affected by strenuous exercise. In this study, the influence of this factor on the thickness of the knee cartilage was reduced by avoiding strenuous exercise from the evening before the MRI examination, taking into account previous studies. In addition, it was found that the thickness of articular cartilage at the medial femoral condyle and medial and lateral tibial plateaus tended to thin with age in normal adults aged 20–40 years in China, but there was no corresponding thinning of patellar cartilage. Due to the limited sample size and short follow-up time of this experiment, the contralateral healthy patellar cartilage was not included in the observation subjects. Due to the limited measurement method, this experimental study did not assess the changes in thickness of the entire patellar cartilage, and the small sample size and relatively short follow-up period of this experimental study limited the persuasiveness of the experimental results. Further studies could expand the sample size and provide continuous observation and comprehensive measurement of bilateral patellar cartilage thickness in patients with ACL reconstruction over a long follow-up period in time.

The main findings of this experimental study were a decrease in patellar cartilage thickness and an increase in ISR at 6-month follow-up after anterior cruciate reconstruction compared with that before reconstruction, and the differences were statistically significant, as shown in Figure 4. The decrease in patellar cartilage thickness after ACL reconstruction may be related to the occurrence and development of patellar cartilage injury and patellofemoral osteoarthritis after ACL reconstruction, and the related mechanism still needs further investigation. The increase in ISR after ACL reconstruction compared with that before reconstruction may be caused by the recovery of patellar tendon morphology from tortuous shortening after ACL reconstruction, given the high incidence of patellofemoral cartilage damage and patellofemoral osteoarthritis after ACL reconstruction. Therefore, tracking changes in patellofemoral cartilage thickness in patients after ACL reconstruction is important for the early diagnosis and intervention of patellofemoral cartilage injury and degeneration in patients after reconstruction, as well as for the prevention of the occurrence and development of patellofemoral osteoarthritis.

### 3.3. Meniscal Injury and Inflammation

Patients with ACL injuries often have combined meniscal injuries, and studies have demonstrated that combined meniscal injuries found during ACL reconstruction are an independent risk factor for postoperative osteoarthritis of the knee. Further experiments have found that meniscectomy in patients with ACL injury predicts the development of postoperative patellofemoral arthritis. A 10-year follow-up of patients after ACL reconstruction revealed that meniscectomy was an important risk factor for the development of patellofemoral arthritis after surgery. Similarly, a mathematical model using information obtained at a 6-year follow-up after reconstructive surgery identified meniscectomy at the time of reconstruction as a significant predictor of postoperative patellofemoral arthritis. It has also been shown that removal of the knee meniscus can have an effect on the horizontal rotational function of the tibiofemoral interarticular joint, and this effect is more pronounced during exercise, as shown in Figure 5. It was found that a tear of the posterior horn of the medial meniscus in a cruciate ligament-injured knee would increase relative tibiofemoral rotation. These changes in tibiofemoral relative rotation, in turn, affect the contact stresses in the patellofemoral joint, reducing the thickness of the patellofemoral cartilage. Although no studies have evaluated patellofemoral joint alignment after meniscectomy, changes in frontal plane moments of the patellofemoral joint have been observed after partial meniscectomy compared to healthy controls. Based on the above studies, it can be partially explained how the patellofemoral joint is affected after meniscectomy, but further studies are still needed. Based on the results of the current study, it can be inferred that maximizing meniscal preservation during ACL reconstruction may reduce the incidence of postoperative patellofemoral arthritis.

During the acute phase of ACL trauma, the initiation of cellular inflammatory factors and protease cascade reactions hydrolyze the network of protein molecules in the articular cartilage, which erodes the articular cartilage and may lead to degeneration of patellofemoral cartilage. It has been shown that numerous cellular inflammatory factors may often be present for a considerable period of time after ACL injury before finally tapering off. In addition, the surgical operation itself is an irritant that inevitably prolongs the inflammatory response of the joint or creates new inflammation. Cellular inflammatory factors, degradative enzymes, and cartilage breakdown products in the synovial fluid at the time of ACL reconstruction have been noted as important predictors of knee cartilage degeneration at the third-year postoperative follow-up. However, although there was more cartilage damage in the knee 8 years after ACL reconstruction, the levels of inflammatory cytokines and biomarkers were not significantly different compared to the healthy knee. There is conflicting evidence from the above studies and further studies are awaited. The current possible explanation is that while these inflammatory responses may be associated with early articular cartilage degeneration after ACL reconstruction, they are not a major factor in the development of distant articular cartilage degeneration.

## 4. Results and Discussion

Anterior cruciate ligament injury is a common clinical condition, mostly caused by strenuous sports or accidental injury, which is also related to its anatomical structure. Trauma-induced ACL rupture can be accompanied by medial collateral ligament and medial meniscus injury, which can seriously affect the stability of the knee joint. In most patients, conservative treatment is ineffective and can lead to joint instability and degeneration. Therefore, early, noninvasive, and accurate diagnosis of ACL injuries is essential in clinical practice. Arthroscopy is the gold standard for the diagnosis of ACL injury, and this technique has both clinical roles of examination and treatment, which can effectively target the injury site for repair and treatment and can also accurately find the lesion site and determine the degree of ligament injury through visual and three-dimensional observation for ligament injuries that are difficult to detect on imaging. In this paper, we performed MPR and VRT on patients with ACL injury and postprocessed the data. The diagnostic compliance rate of dual-source CT was 91.67% (33/36), the true-positive rate was 93.33% (28/30), the missed rate was 6.67% (2/30), and the true-negative rate was 83.33% (5/6). The rate of true negative was 83.33% (5/6), and the rate of false diagnosis was 16.67% (1/6). Kappa analysis of the consistency between dual-source CT and arthroscopy showed a Kappa value of 0.719, indicating a high degree of consistency between the two examination methods. In conclusion, MPR and VRT images are of clinical value for the diagnosis of ACL injury. The clinical applications of MPR and VRT are widely used, not only in the postprocessing reconstruction of soft tissues, but also in the diagnosis of bone diseases. Although the principles of MPR and VRT imaging are not discussed in detail in this paper, their important clinical role is well recognized and will not be repeated here. The mean CT values of the affected side of the ACL and the normal side of the ACL were (63.52 ± 2.97) Hu and (70.99 ± 4.26) Hu, respectively, as shown in Figure 6. As shown in Figure 6, the CT values of all patients with ACL injury were measured to be lower than those of the normal side, and the CT values of complete ligament rupture were most significantly reduced, which may be related to periligamentous edema or exudation.

The thickness values of the segments of the ACL on the normal side were (4.00 ± 0.02) mm, (3.76 ± 0.04) mm, and (3.94 ± 0.03) mm, and the thicknesses of the beginning and end segments were slightly greater than those of the middle segment, which was consistent with the normal anatomy of the ACL, as shown in Figure 7, while the thicknesses of the ACL region of interest on the affected side increased to different degrees, and the thickening of the beginning and middle segments was the most significant. The thickness of the ACL zone of interest on the affected side increased to different degrees, and the thickening of the beginning and middle segments was the most obvious. The *t*-test of the thickness of the thickened segment on the affected side and the normal side showed that the values obtained were *P* < 0.05, and the differences were statistically significant. When the changes in the length of the anterior cruciate ligament were analyzed bilaterally, the length values of the normal side and the affected side were (29.84 ± 1.55) mm and (29.40 ± 41.34) mm, respectively, and the obtained values were *P* < 0.05, indicating that the length of the affected side was shorter than that of the normal side, which was statistically significant, and the analysis may be due to the contracture of the ligament caused by partial or complete tear of the ligament (Figure 8).

In summary, the CT values of the anterior cruciate ligament and the thickness of each segment can be measured by the MPR and VRT imaging techniques of dual-source CT for the diagnosis of injury, which is based on specific numerical changes and has a certain degree of objectivity. 26 of the 30 cases of arthroscopically confirmed anterior cruciate ligament injury showed reduced or absent dual-energy staining, and 4 cases showed no significant change in dual-energy staining. This is similar to previous findings. In the four cases with no significant change in dual energy staining, the arthroscopic examination showed a mild partial tear of the ligament. The cause of the change in dual-energy staining of the ligament was associated with changes in the content of dense hydroxylysine and hydroxyproline, and further observation of the cause and association is needed in future studies. In conclusion, dual-source CT can diagnose ligament injury in an objective, quantitative, and noninvasive manner by measuring the CT values of the anterior cruciate ligament and the thickness of each segment through MPR and VRT postprocessing techniques and can predict ligament injury in a more intuitive manner using dual-energy staining techniques, which is not available in some arthroscopes. Therefore, combined with the results of our above analysis, we conclude that the postprocessing application of dual-source CT images can be used as an important imaging aid for the diagnosis of ACL injury; the initial diagnosis and localization of ACL injury can be made by dual-source CT imaging measurements.

## 5. Conclusion

The mean CT values of the affected and normal sides of the ACL were (63. 52 ± 2. 97) Hu and (70. 99 ± 4. 26) Hu, respectively, and the CT values of all patients with ACL injuries were lower than those of the normal side. The CT values of all patients with anterior cruciate ligament injury were lower than those of the normal side, and the CT values of complete ligament rupture were most significantly reduced, which may be related to periligamentous edema or exudation. The results suggest that abnormal patellofemoral joint biomechanics may lead to patellofemoral joint cartilage degeneration, which may further lead to patellofemoral joint osteoarthritis, since normal cartilage mechanical loading is essential for cartilage development and maintenance. CT examination has a higher soft tissue resolution compared to other tests and can scan the damaged area from multiple angles, and the difference in MRI images between partial and complete tears of the anterior cruciate ligament of the knee is significant. The difference in imaging is significant, so there is a clear advantage in identifying more accurately whether the ACL fibrous elements are intact.

## Figures and Tables

**Figure 1:** Complications in ACL reconstruction.

**Figure 2:** Association of patellar cartilage damage after anterior cruciate ligament reconstruction.

**Figure 3:** Anterior displacement of tibia relative to femur.

**Figure 4:** Change in patellar cartilage thickness compared to prereconstruction.

**Figure 5:** Meniscal injury at CT.

**Figure 6:** CT values of patients with ACL injury compared to normal side CT values.

**Figure 7:** ACL thickness values by segment.

**Figure 8:** Changes in dual-energy staining.

**Table 1:** The general information of selected patients.

Group	Average age (years old)	Gender (male/female)	Course of disease (month)	Injury part	
				Left	Right
Control	33.5 ± 10.8	21/15	2–13	18	22
Observation	35.2 ± 12.5	21/15	2–13	18	22

## Data Availability

The data used to support the findings of this study are available from the corresponding author upon request.
